The article "GINS2 Is Downregulated in Peripheral Blood of Patients with Intervertebral Disk Degeneration and Promotes Proliferation and Migration of Nucleus Pulposus Cells" was retracted in 2023. Reasons: signs of a paper mill; compromised peer review; unreliable results or conclusions.

# GINS2 Is Downregulated in Peripheral Blood of Patients with Intervertebral Disk Degeneration and Promotes Proliferation and Migration of Nucleus Pulposus Cells

**DOI:** 10.1155/2022/1986348

**Published:** 2022-09-01

**Authors:** Haitao Jiang, Hailang Sun, Jian Dai, Cheng Zhang, Xiaoming Tang

**Affiliations:** Department of Orthopedics, The Affiliated Huaian No.1 People's Hospital of Nanjing Medical University, Huai'an, 223300 Jiangsu, China

## Abstract

GINS complex subunit 2 (GINS2) regulates the migration, invasion, and growth of cells in many malignant and chronic diseases. In the present study, we aimed to investigate the expression of GINS2 in the peripheral blood and nucleus pulposus (NP) cells of patients with intervertebral disk degeneration (IDD). GINS2 expression was detected using bioinformatics tools from the GEO public repository and validated using peripheral blood samples from IDD patients and healthy participants. GINS2 clinical significance was explored by the receiver operating curve (ROC) utilizing area under the curve (AUC). Moreover, the influences of GINS2 on cell viability, migration, and invasion were explored by MTT, wound healing, and transwell assays, whereas cell apoptosis was determined by flow cytometry. Expression levels of GINS2 in the peripheral blood were significantly lower in IDD patients than in healthy participants. Moreover, ROC obtained a significantly higher AUC of GINS2 in IDD patients. Further, overexpressed GINS2 increased the proliferation, migration, and invasion of NP cells while overexpressed GINS2 decreased the apoptotic property of cells compared to the NC plasmid and control groups. In conclusion, GINS2 might be a potential therapeutic target of IDD.

## 1. Introduction

Intervertebral disk degeneration (IDD) is a leading factor of discogenic lower back pain (LBP) [1–3]. IDD has been relegated to the disc tissue-based age-related process due to the continuously decreasing concentration of proteoglycan, which leads to decreased intervertebral height, the production of osteophytes, and endplate sclerosis [4, 5]. A normal human intervertebral disc is a fibrocartilaginous structure made of three main components, such as (1) cartilage endplates [6, 7]; (2) the annulus fibrosus (AF), composed of type I collagen and fibroblast-like cells [8]; and (3) nucleus pulposus (NP) originated of chondrocyte-like cells [9, 10]. Previous studies have found that the inherited factors were directly linked to the pathogenic factors (almost 70%) that were associated with IDD [11–13]. Thus, assessing the IDD mechanism from a genetic standpoint is crucial to address the present clinical concerns about chronic LBP.

GINS complex subunit 2 (GINS2), a member of the GINS family that also includes GINS2, GINS3, and GINS4 [14], plays an essential role in the DNA duplication [15]. Downregulation of GINS2 suppressed the growth of breast cancer cells by triggering endogenous DNA damage [16, 17]. Further, a study reported that unregulated expression of GINS2 initiated free survival of distant metastasis and therapeutic resistance of endocrine in patients with breast cancer [18]. Meanwhile, upregulated GINS2 urged the proliferation of HL60 cells in acute promyelocytic leukemia [19]. Moreover, overexpressed GINS2 promoted cell migration and proliferation and repressed apoptosis in lung cancer cell lines [20]. Nonetheless, the role of GINS2 in the peripheral blood and NP cells of patients with intervertebral disk degeneration (IDD) remains unknown.

In this study, we found that GINS2 was downregulated in the peripheral blood and NP cells of IDD patients and had a significant diagnostic value for IDD. Moreover, we confirmed the promotive effects of GINS2 overexpression on the proliferation, migration, and invasion and the inhibitory effect on the apoptosis of NP cells. Our study might provide a novel target for IDD therapy.

## 2. Materials and Methods

### 2.1. Study Design

The present study is aimed at evaluating the GINS2 protein-coding gene expression using a GEO-based repository and further validates it retrospectively in the peripheral blood samples of IDD patients and healthy participants. Subsequently, the expression of GINS2 was achieved in IDD patients. Finally, GINS2 expression and its biological functions were analyzed in vitro using NP cells.

### 2.2. Enrollment of Patients

60 participants with IDD (*n* = 30) and healthy control (*n* = 30) were retrospectively collected, along with the peripheral blood samples. The subjects were enrolled from June 2020 to June 2021.

### 2.3. Cell Culture and Cell Transfection

Human NP cells (CP-H170, Procell, Hubei, China) were used in the present study. Herein, cells were cultured in Roswell Park Memorial Institute (RPMI-1640) medium (Thermo Fisher Scientific, MA, USA) comprising 10% fetal bovine serum (FBS, Gibco, NY, USA) and penicillin in a 37°C and 5% CO_2_ incubator. Furthermore, the cells were seeded onto a 12-well plate. GINS2-overexpression (GINS2-OE) plasmid, negative control (NC) plasmid, and blank control were transfected into NP cells by Lipofectamine 300 (Invitrogen, CA, USA) for 48 h. They were bought from GenePharma Biotechnology Co. Ltd., (Shanghai, China). Then, all the cells were obtained and utilized for subsequent experiments.

### 2.4. RNA Extraction

Total RNA was isolated from the whole blood cells of the peripheral blood samples utilizing phenol-chloroform solutions after handling the homogenization by guanidine isothiocyanate (kit for preparing TRIzol RNA, Thermo Fisher Scientific, Waltham, MA, USA). RNA concentrations were analyzed by a spectrophotometer (ND1000, NanoDrop Technologies, DE, USA).

### 2.5. RT-qPCR

Total RNA was isolated from the peripheral blood specimens by following TRIzol reagent protocols after transfection. Then, using the reverse transcript kit, the total RNA was reverse-transcribed to cDNA (Sangon Biological Engineering Co., Shanghai). Reaction steps of qPCR were carried out using SYBR Green PCR Master Mix (Applied Biosystems, USA) as follows: (1) for 10 min at 95°C (predenaturation); (2) for 15 s at 95°C (denaturation), for 15 s at 60°C (annealing), and for 20 s at 72°C (elongation); and (3) for 15 min at 72°C. At 4°C, reactions were discontinued. For each specimen, these three steps were followed, and a quantitative analysis of the data was performed based on a 2^−△△CT^ value. The RT primers utilized were as follows: GINS2, forward: 5′-AGGCGCCAGAGGCACCATGGAC-3′ and reverse: 5′-CATCCTGTGCGTTGGCTGCC-3′; *β*-actin, forward: 5′-GAGCGCGGCTACAGCTT-3′ and reverse: 5′-TCCTTAATGTCACGCACGATTT-3′.

### 2.6. Microculture Tetrazolium (MTT) Assay

MTT assay was carried out to evaluate the proliferation activity of the cell by following the manufacturer's protocols (Beyotime Biotech., Shanghai, China) [21]. NP cell lines were cultivated in 96-well plate at 5 × 10^3^ cells/well density and then treated with overexpression of the GINS2 plasmid. 10 *μ*L MTT reagent (Beyotime Biotech., Shanghai, China) was imparted into the well and further incubated for 4 h at 37°C. Each well's optical density (OD) value was evaluated by a microplate reader (Promega Corporation, Madison, WI, USA) at 490 nm. Results of the cell viability from three independent experiments were normalized to the control group and expressed as mean ± SD.

### 2.7. Transwell Assay

Matrigel was equally spread on the transwell chamber's bottom surface (Corning, Shanghai, China). After 10% FBS, 500 *μ*L medium was put into the lower chamber, and 2 × 10^4^ cells were added to the upper chamber. Then, cells on the upper surface were gently scraped, whereas the invasive cells on the lower surface were fixed and colored with crystal violet, followed by observation using a microscope (Olympus Corporation, Tokyo, Japan).

### 2.8. Wound Healing Assay

After the transfection of NP cells, the cells were treated with trypsin, planted into the 6-well plate, and cultivated till they reached 80% confluence of the medium. Then, the sterile pipette (200 *μ*L) tip was used to scratch each well and washed with PBS solution numerous times to abolish cell debris. In the following 48 h, cells were incubated in medium (serum-free), and migrated cells to the surface of the wound were counted as fabricating an in vitro healing process. The display images of the wound healing assay were obtained by a light microscope (Olympus Corporation, Tokyo, Japan; magnification ×100), and the closure rate was evaluated. The relative ability of migratory cells was assessed by ImageJ software using the width at 0 h time point ((width of wound (0 − 24 h)/0 h width of wound) × 100%).

### 2.9. Apoptosis Assay

The cells were put into a 12-well plate after transfection, and NP cells were obtained from trypsin digestion without EDTA (Thermo fisher, Waltham, MA, USA). The rate of apoptotic cells was evaluated by Annexin V-PE/7-AAD (Sungene Biotech., Tianjin, China) following the manufacturer's protocols and instructions. Herein, cells were stained using 5 *μ*L Annexin V-phycoerythrin (PE) and 5 *μ*L 7-amino-actinomycin D at 37°C for 10 min. The cells were determined by flow cytometry (BD Aria III, New Jersey, USA).

### 2.10. Western Blotting

After 48 h posttransfection, the cells were kept in a 6-well plate and managed under suitable conditions. After the cells were put into the RIPA assay buffer (Beyotime Biotech., Shanghai, China), protein in equal amounts was parted by SDS-PAGE and transferred onto PVDF membranes (Bio-Rad, CA, USA). Then, the membranes were blocked with skim milk (5%), cleansed with Tris-buffered saline, and incubated with primary antibodies, GINS2 (1 : 200, ab197123, Abcam, MA, USA) and GAPDH (1 : 1000, 5174T, Cell Signaling Technology, MA, USA), overnight at 4°C. After that, the membranes were incubated with secondary antibody HRP-conjugated goat antirabbit IgG heavy and light (1 : 2000, ab6721, Abcam) for 1 h. Furthermore, the membranes were analyzed by an ECL reagent (Thermo Scientific Pierce, IL, USA). The protein band was visualized with the internal reference of *β*-actin.

### 2.11. Bioinformatics and Statistical Analysis

Bioinformatics tools were used to create box plots, PCA biplots, volcano maps, and heatmaps. By utilizing the GEO database (GSE124272), the enriched signaling pathways were evaluated through the Kyoto Encyclopedia of Genes and Genomes (KEGG) and Gene Ontology (GO) databases. GraphPad (version 8, CA, USA) and SPSS software (version 20.0, IL, USA) were used for statistical analysis throughout the study, and all the data were represented as mean ± standard deviation. *T*-test and one-way and two-way ANOVA analyses were utilized to compare two or more groups. GINS2 clinical significance was explored using the receiver operating curve- (ROC-) based area under the curve (AUC) in the peripheral blood samples. *P* < 0.05 was contemplated as the threshold for providing statistical significance.

## 3. Results and Discussion

### 3.1. Discovery of GINS2 Expression in IDD

Eight microarray datasets of IDD patients compared to healthy controls were obtained from the GEO database (GSE124272) and used to screen for the GINS2 protein-coding gene utilizing bioinformatics tools, resulting in dysregulated gene expressions as determined by box plot, PCA biplot, volcano map, and heatmap analyses (see Figures 1(a)–1(d)). These eight datasets have demonstrated GINS2 expressions individually (see Figure 2(a)). PCA biplots were shown as the quantitative measure of eight microarray datasets (see Figure 2(b)). Based on these biplots of PCA, the present study involved all eight datasets for subsequent analysis. In the box plot, GINS2 expressions were significantly lower in IDD patients contrasted to a healthy group (see Figure 2(c), *P* < 0.05).

Moreover, the top 20 significant KEGG pathway enrichments in IDD patients and healthy groups based on the up- and downregulated genes were obtained utilizing the KEGG database (see Figure 3(a), *P* < 0.05). Likewise, significant top 20 GO enriched pathways related to the up- and downregulated genes were achieved using the GO database (see Figure 3(b), *P* < 0.05).

### 3.2. Validation and Clinical Significance of GINS2 in IDD Patients

To validate GINS2 expression levels in the peripheral blood from 30 IDD patients and 30 healthy participants, a scatter plot analysis was used. Herein, GINS2 expression was markedly decreased in the peripheral blood samples of IDD patients compared to the healthy group (see Figure 4(a), *P* < 0.001). Meanwhile, the demographical parameters of IDD patients and healthy participants are represented in Table 1, which showed no significant differences (*P* > 0.05). The ROC curve of GINS2 yielded a significantly high AUC of 0.8261 (95% confidence interval (CI) = 0.7051 ~ 0.9472, *P* < 0.05) in IDD patients (see Figure 4(b)). Thus, the diagnostic values of GINS2 may be used to precisely distinguish between IDD patients and healthy groups and further provide potential significance in diagnosing IDD.

### 3.3. Cell Proliferation, Migration, and Invasion Effects of GINS2 in NP Cells

The present study evaluated the biological functions of GINS2 by transfecting NP cells with the GINS2-OE and NC plasmids. WB analysis was utilized to determine the expression of GINS2 mRNA in NP cells transfected with NC plasmid, blank group, and GINS2-OE plasmid (see Figures 5(a) and 5(b), *P* < 0.001). GINS2 mRNA expression was significantly over/upregulated in NP cells following transfection with the GINS2-OE group compared to other groups (*P* < 0.001). Similarly, the CCK-8 assay demonstrated that the overexpression of GINS2 markedly increased cell viability (see Figure 5(c), *P* < 0.001), indicating that GINS2 upregulation may promote the proliferation of NP cells.

The migration and invasion abilities of cells are key indicators of tumor metastasis. The current study utilized wound healing and transwell assays to detect the metastatic capability of the tumor. Wound healing assay showed that the GINS2-OE significantly increased and promoted the migratory potential of NP cells when compared to the NC plasmid and blank groups (see Figures 5(d) and 5(e), *P* < 0.001). Subsequently, a transwell assay was utilized to determine the invasive ability of NP cells, which showed that GINS2-OE significantly promoted the invasion capability of NP cells when compared to other groups (see Figures 6(a) and 6(b), *P* < 0.001). Hence, the overexpression of GINS2 could promote NP cell migration and invasion.

### 3.4. Cell Apoptosis Effects of GINS2 in NP Cells

To determine the apoptosis effects of GINS2 in NP cells, Annexin V-PE/7-AAD staining was utilized. The apoptosis assay demonstrated that GINS2-OE significantly decreased the apoptosis rate in NP cells when compared to the NC plasmid and blank groups (see Figures 7(a)–7(d), *P* < 0.001). Thus, overexpression of GINS2 inhibited NP cell apoptosis.

## 4. Discussion

IDD is widely recognized as a major cause of LBP, a globally prevalent condition that imposes a vast social-economic burden and degrades the quality of life [22–24]. Disk degeneration is also associated with disk prolapse or herniation and sciatica, though it can be asymptomatic in some cases [25, 26]. In IDD cases, the intervertebral disk height and spinal column-based biomechanics are altered, which can have a significant effect on the behavior of other spinal structures, involving the ligaments and muscles [7]. In the long run, this condition can progress to spinal stenosis [27], which is the main reason for pain and disability in the aged population [25]. Overall, IDD is a tangled process whose mechanism is not fully apprehended. Extracellular matrix degeneration, mechanical loading, extreme senescence, incremental secretions of inflammatory factors, and NP cell aberrant apoptosis have all been implicated in the development of IDD [28–32]. Thus, current research into NP cell apoptosis and targeted interventions may not only anticipate significant therapeutic strategies but also increase the underlying pathogenetic mechanisms of IDD.

GINS2 takes a crucial part in the replication activity and chromatin binding due to the complex structure as a heterotetramer [33]. In malignant cancers, such as cervical cancer, GINS2 was significantly upregulated in cancer cells and tumor tissues with an inverse correlation to overall survival in cervical cancer patients [34], whereas in thyroid cancer, GINS2 overexpression initiated the cancer cell proliferation and suppressed the apoptosis via LOXL2 and CITED2 mediation [35, 36]. Our study determined and confirmed the dysregulation of GINS2 expression in the peripheral blood samples from IDD patients and healthy participants. Our pathway enrichment analysis results indicated that GINS2 was involved in KEGG-enriched pathways, including p53 signaling pathways, cell cycles, extracellular matrix, and cytokine receptor interactions in IDD-based samples. Hence, on one hand, GINS2 was demonstrating downregulated expression in the peripheral blood samples from IDD, and on the other hand, GINS2 may take part in IDD pathogenesis via certain enriched pathways. Moreover, our study indicated that GINS2 protein-coding gene significantly differentiated IDD patients from the healthy group by representing an AUC of 0.8261. Thus, GINS2 protein-coding gene not only played a role in IDD pathogenesis but may also serve as a novel diagnostic biomarker for IDD by distinguishing IDD patients from healthy controls.

GINS2 was previously shown to influence the proliferation, migration, and invasion of non-small-cell lung cancer cells via PI3K/Akt and MEK/ERK signaling pathways [37]. Similarly, interfering with GINS2 inhibited cell viability, initiated cell cycle arrest, and facilitated apoptosis in pancreatic cancer cell lines using the MAPK/ERK pathway [38]. Our study evaluated the biological functions of GINS2 in NP cells by GINS2-OE and NC plasmids. Herein, consistent with the above-mentioned studies, our in vitro analysis revealed that the overexpression of GINS2 promoted cell proliferation, migration, and invasion of NP cells; meanwhile, it suppressed the apoptotic activity and vice versa. Thus, GINS2 may act as a potential therapeutic target for IDD.

Nonetheless, the current study has a few limitations. At first, the determination of GINS2 was screened using an online database of GEO, which could contain biased microarray results or samples. Second, GINS2 validation was carried out with a smaller size-based cohort; therefore, future studies are needed to carry out validation using a larger size-based cohort. Third, the present study was unable to include more clinical characteristics and risk factors for patients with IDD. Fourth, the GINS2 was evaluated and compared using only the peripheral blood samples and NP cell lines without further validation of downregulating signaling pathways. Thus, future research is required to thoroughly determine and assess GINS2 in conjunction with other GINS family members, which might be taking part in the occurrence, development, and progression of IDD.

## 5. Conclusion

In conclusion, downregulation of GINS2 was observed in the peripheral blood and NP cells of IDD patients, which had a significant diagnostic value for IDD. Moreover, our study proved GINS2 overexpression promoted the proliferation, migration, and invasion and inhibited the apoptosis of NP cells, implying the biological role of GINS2 in IDD. GINS2 might be a novel target for IDD therapy.

## Figures and Tables

**Figure 1:** Screening of the genes between IDD patients and healthy control group. (a) The expression value of multiple genes shown in IDD patients versus healthy control by each of the eight microarray datasets of the GEO database (GSE124272) in the box plot. (b) PCA biplots of eight microarray datasets represented quality control measures. (c) Volcano plot is representing the dysregulated expression of genes. (d) Heatmap is showing the up- and downregulated expressed genes between two groups.

**Figure 2:** Discovery of the GINS2 between IDD patients and healthy control group. (a) The expression value of multiple genes observed in IDD patients versus healthy control by each of the eight microarray datasets of the GEO database (GSE124272) in the box plot. (b) PCA biplots of eight microarray datasets showed quality control measures. (c) GINS2 expression was measured in the peripheral blood from two groups of participants by box plots. G1: healthy group; G2: IDD group.

**Figure 3:** GO and KEGG pathway enrichment analysis. (a) The top significant KEGG-enriched pathways of the targeted genes in IDD are demonstrated individually in up- and downregulated manner. (b) The topmost GO enrichment pathways of the targeted genes in IDD are shown in a similar manner.

**Figure 4:** The validation of GINS2 expression in the peripheral blood samples between IDD patients and healthy control. (a) The histogram represented the overall validation of GINS2 in IDD patients and healthy control. (b) The clinical significance of GINS2 was measured by ROC curve for IDD patients.

**Figure 5:** The biological mechanism of GINS2 in NP cells. (a, b) Western blot analysis represented the GINS2 mRNA expression in three groups of GINS2-OE, NC plasmid, and blank group. (c) MTT assay showed the cell proliferation or growth rate of three groups in transfected NP cells. (d) The wound healing rate was observed between the three groups. (e) Wound healing assay was performed to evaluate the migratory ability of transfected NP cells. NC plasmid, blank group, and GINS2-OE.

**Figure 6:** Effects of GINS2 on migration and invasion of NP cells. (a, b) Transwell assay was performed on NP cells and showed the invasive capacity of cells. NC plasmid, blank group, and GINS2-OE.

**Figure 7:** The apoptosis assay of NP cells. (a–d) NP cells transfected with GINS2-OE, NC plasmid, and blank group showed the apoptotic activity of cells.

**Table 1:** Clinical information of the patients and healthy controls.

	Control (*n* = 30)	IDD (*n* = 30)	*P* value
Age (years)	35.14 ± 4.21	36.22 ± 4.95	0.1166
BMI	24.31 ± 2.35	25.06 ± 2.78	0.0522
Gender (male/female)	18/12	11/19	0.8586

## Data Availability

The datasets used during the current study are available from the corresponding author on request.
